The article "Establishment and Validation for Predicting the Lymph Node Metastasis in Early Gastric Adenocarcinoma" was published in 2022. Journal: J Healthc Eng.

# Establishment and Validation for Predicting the Lymph Node Metastasis in Early Gastric Adenocarcinoma

**DOI:** 10.1155/2022/8399822

**Published:** 2022-06-29

**Authors:** Xuan Li, Haiyan Zhou, Xianhui Zhao, Huan Peng, Shanshan Luo, Juan Feng, Jianfu Heng, Heli Liu, Jie Ge

**Affiliations:** ^1^Department of Gastrointestinal Surgery, Xiangya Hospital, Central South University, Changsha 410008, Hunan, China; ^2^Department of Pathology, Xiangya Hospital, Central South University, Changsha 410008, Hunan, China; ^3^Department of Clinical Pharmaceutical Research Institution, Hunan Cancer Hospital, Affiliated Tumor Hospital of Xiangya Medical School of Central South University, Changsha 410008, Hunan, China; ^4^The Hunan Provincial Key Laboratory of Precision Diagnosis and Treatment for Gastrointestinal Tumor, Changsha 410008, Hunan, China

## Abstract

Lymph node metastasis (LNM) is considered to be one of the important factors in determining the optimal treatment for early gastric cancer (EGC). This study aimed to develop and validate a nomogram to predict LNM in patients with EGC. A total of 842 cases from the Surveillance, Epidemiology, and End Results (SEER) database were divided into training and testing sets with a ratio of 6 : 4 for model development. Clinical data (494 patients) from the hospital were used for external validation. Univariate and multivariate logistic regression analyses were used to identify the predictors using the training set. Logistic regression, LASSO regression, ridge regression, and elastic-net regression methods were used to construct the model. The performance of the model was quantified by calculating the area under the receiver operating characteristic curve (AUC) with 95% confidence intervals (CIs). Results showed that T stage, tumor size, and tumor grade were independent predictors of LNM in EGC patients. The AUC of the logistic regression model was 0.766 (95% CI, 0.709–0.823), which was slightly higher than that of the other models. However, the AUC of the logistic regression model in external validation was 0.625 (95% CI, 0.537–0.678). A nomogram was drawn to predict LNM in EGC patients based on the logistic regression model. Further validation based on gender, age, and grade indicated that the logistic regression predictive model had good adaptability to the population with grade III tumors, with an AUC of 0.803 (95% CI, 0.606–0.999). Our nomogram showed a good predictive ability and may provide a tool for clinicians to predict LNM in EGC patients.

## 1. Introduction

Gastric cancer, the third leading cause of cancer death in the world, is responsible for more than 1 million new cases each year [1]. Morbidity and mortality of gastric cancer were higher in East Asia, East Europe, and South America [2–5]. In addition, approximately half of the estimated deaths from gastric cancer in 2018 occurred in China [1]. Early gastric cancer (EGC) is defined as gastric cancer confined to the lamina propria or mucosa and submucosa, regardless of the size or presence of regional lymph node metastasis (LNM) [6]. LNM is the most common form of gastric cancer metastasis and a major contributor to the high mortality. In the TNM staging system of gastric cancer, LNM was used to guide the treatment plan, and the prognosis was predicted by the number of pathologically positive lymph nodes and the exact stage of the disease [7].

The main treatment methods for EGC include endoscopic mucosal resection (EMR) or endoscopic submucosal dissection (ESD), wedge resection, laparoscopically assisted gastrectomy, and open gastrectomy [8, 9]. Compared with other treatment methods, EMR and ESD can preserve gastric function and maintain quality of life [10, 11]. However, the absence of LNM is a prerequisite for EMR and ESD [12]. Therefore, a tool that can predict LNM in EGC patients was of great significance for surgical methods selection and of patients' prognosis. Several studies have established nomograms for LNM in patients with EGC [6, 13, 14]. However, these studies had some limitations, such as small sample size, single-center research, and no external validation. In addition, there were few studies on the predictive effect of LNM on EGC patients in different populations.

Herein, we selected the predictor variables of LNM in EGC patients based on the Surveillance, Epidemiology, and End Results (SEER) database. Then, a nomogram to predict the LNM in EGC patients was developed, and external validation was performed to assess the fit of the model.

## 2. Methods

### 2.1. Study Design and Population

Data were extracted from the SEER database, which is a national sample of the population-based cancer database proposed by the National Cancer Institute. The SEER database covers approximately 28% of the entire American population. All patients with gastric adenocarcinoma were extracted from the SEER database from 2015 to 2020. For external validation, 494 patients who had been diagnosed with EGC were collected from the Xiangya Hospital Center South University between January 2012 and December 2019. Tumors were staged based on the criteria of the American Joint Committee on Cancer (AJCC) Staging Manual (7th), and EGC in this study included Tis, T1a, and T1b [15]. This study was approved by the Institution Review Board of the Xiangya Hospital Center South University (approval number: 2019030510), and all patients provided written informed consent.

### 2.2. Inclusion and Exclusion Criteria

Patients who met the following inclusion criteria were eligible for inclusion: (1) patients' age ≥18 years; (2) patients who were diagnosed by histopathology as stage Tis, T1a, or T1b gastric adenocarcinoma; (3) patients with complete baseline data and pathological data. The exclusion criteria were as follows: (1) patients with no surgical resection or microscopic evaluation of lymph nodes; (2) patients who received radiotherapy or chemotherapy before surgery; (3) patients with metastasis at the time of diagnosis; (4) patients with other gastric tumors (neuroendocrine, gastrointestinal stromal tumors or metastatic disease); (5) patients with a history of other malignancies.

### 2.3. Data Collection

Demographic and clinical data included the patient's age, gender, T stage, primary site, tumor size, tumor grade, and LNM. The tumor stage was assigned to Tis, T1a, and T1b stages. Tumor size was divided into <1 cm, 1-2 cm, 2-3 cm, 3-4 cm, and ≥4 cm. LNM was used as an outcome indicator.

### 2.4. Statistical Analysis

Data were extracted from the SEER database using SEER^*∗*^Stat data retrieval software (version 8.3.2). The data were divided into the training set and test set in a 6 : 4 ratio. The clinical practice data were used for external validation. Continuous variables with normal or approximately normal distribution were expressed as mean ± standard deviation (SD), and a *t*-test was used for comparison between groups. Nonnormal variables were expressed as M (Q1, Q3), and the Wilcoxon rank-sum test was used for comparison between groups. Categorical variables were expressed in numbers and percentages, and the Chi-square test (*χ*^2^) or Fisher's test was used for comparison between groups.

Univariate analysis and multivariate logistic regression analysis were used to select prediction variables and establish the prediction model. Logistic regression, LASSO regression, ridge regression, and elastic-net regression methods were used to construct the model. Meanwhile, the nomogram of the prediction model was drawn, and the Hosmer-Lemeshow goodness of fit test was performed on the predictive model. The performance of the model was quantified by calculating the area under the receiver operating characteristic curve (AUC) with 95% confidence intervals (CI), as well as sensitivity, specificity, positive predictive value (PPV), and negative predictive value (NPV).

All statistical analyses and drawings were carried out using the R software (version 4.0.2). The caret package was used to normalize the data, and the relevant parameters for modeling were lambdas <-seq (0.0001, 0.01, length. out = 200). The glmnet package was utilized to construct the LASSO regression, ridge regression, and elastic-net regression models, and threefold cross-validation was performed. Others R packages such as compareGroups, ResourceSelection, rms, and pROC were also used. All tests were two-sided, and the test level was *α* = 0.05.

## 3. Results

### 3.1. Baseline Characteristics

Totally, 842 cases from the SEER database and 494 cases from clinical practice were included in this study (Figure 1). Among these 842 patients, the mean age was 69.4 ± 11.3 years, with 485 (57.60%) patients being males. The primary location of the tumor was mostly the lower part of the stomach (54.04%) and the middle part of the stomach (35.99%). The numbers of patients with LNM in the SEER database and clinical dataset were 176 (20.9%) and 133 (26.92%), respectively. More detailed characteristics were shown in Table 1.

### 3.2. Differences in Characteristics of Patients with and without LNM

Table 2 shows the characteristics of patients with and without LNM. The results indicated the significant differences between patients with and without LNM in T stage, tumor size, and tumor grade (all *P* < 0.001). The incidence of LNM was higher in T1b stage patients than in T1a patients (*P* < 0.001). LNM was more likely to occur in tumors larger than 2 cm than in smaller tumors (*P* < 0.001). Tumor grade higher II grade was associated with higher LNM (*P* < 0.001).

### 3.3. Factors Associated with LNM in EGC Patients

The univariate and multivariate logistic regression analyses were shown in Table 3. The multivariate logistic regression analysis indicated that T stage, tumor size, and tumor grade positively were correlated with LNM in EGC patients. The risk of LNM in patients with T1b stage was 3.84 times (OR = 3.84; 95% CI, 2.04–7.21) higher than in patients with T1a stage. Compared with the patients with tumor sizes <1 cm, the risk of LNM in patients with tumor sizes of 2-3 cm, 3-4 cm, and ≥4 cm increased by 2.07 times (OR = 3.07; 95% CI, 1.10–8.61), 3.73 times (OR = 4.73; 95% CI, 1.58–14.13), 4.75 times (OR = 5.75; 95% CI, 2.08–15.92), respectively. The risk of LNM in patients with grade III tumors was 3.19 times (OR = 3.19; 95% CI, 1.27–8.00) higher than in those with grade I tumors.

### 3.4. Model Comparison and Selection

Logistic regression, LASSO regression, ridge regression, and elastic-net regression models were established.  Table 4 presents the AUC of these models in the training set and test set. The AUC of the logistic regression, LASSO regression, ridge regression, and elastic-net regression models in the testing set was 0.766 (95% CI, 0.709–0.823), 0.740 (95% CI, 0.681–0.799), 0.737 (95% CI, 0.676–0.797), and 0.749 (95% CI, 0.691–0.807), respectively. There was no significant difference between the AUCs of these models (*P* > 0.05). The AUC of the logistic regression model was slightly higher than that in the other models, and the results were easier to interpret clinically. Therefore, the logistic regression model was chosen.

### 3.5. Nomogram for Prediction of LNM in EGC Patients

Table 5 displays the performance of the logistic regression model. In the test set, the AUC, accuracy, sensitivity, specificity, PPV, and NPV of the logistic regression model was 0.766 (95% CI, 0.709–0.823), 0.588 (95% CI, 0.533–0.641), 0.899 (95% CI, 0.802–0.958), 0.507 (95% CI, 0.446–0.569), 0.320 (95% CI, 0.255–0.390), and 0.951 (95% CI, 0.902–0.980), respectively. The Hosmer-Lemeshow goodness of fit test showed good calibration (*χ*^2^ = 3.916, *P*=0.917) of this prediction model. However, when external validation was performed using clinical practice data, the AUC of the model was 0.625 (95% CI, 0.537–0.678), implying that the model did not adapt to the external validation data (Figure 2, Table 5).

Then, a nomogram to predict the LNM in EGC patients was drawn based on the logistic regression model. The nomogram can predict the probability of developing LNM in EGC patients by using the sum of the scores determined on the point scale for each variable (Figure 3(a)). An example of the use of this nomogram was as follows: a patient in the SEER database was randomly selected. The patient with the tumor grade III, stage T1b, and tumor size ≥4 cm. The total score of this patient calculated by the nomogram was 243 points, and the possibility of developing LNM was 0.472. After verification, the patient had LNM, and the prediction was successful (Figure 3(b)).

### 3.6. Further Validation Based on Different Populations

Further validation was performed based on gender, age, and tumor grade (Table 6). In the test set, this logistic regression prediction model had a good prediction effect on males, females, patients with age ≥65 years, age <65 years, grade I tumors, and grade III tumors; the AUC of the model in these populations was 0.793 (95% CI, 0.720–0.866), 0.729 (95% CI, 0.635–0.822), 0.755 (95% CI, 0.688–0.821), 0.794 (95% CI, 0.681–0.907), 0.722 (95% CI, 0.583–0.861), and 0.713 (95% CI, 0.647–0.815), respectively. In the external validation data, the prediction model had good adaptability to the population with grade III tumors, with an AUC of 0.803 (95% CI, 0.606–0.999).

## 4. Discussion

In this study, a nomogram for LNM in EGC patients was established based on the SEER database, and external validation was performed by using clinical practice data. Factors associated with LNM in EGC patients such as T stage, tumor size, and tumor grade were included in the nomogram. The AUC, sensitivity, and NPV of the prediction model were 0.766, 0.899, and 0.951, respectively. However, the AUC of the external validation data was 0.625, implying a poor fit for the external population. In addition, further validation was performed based on different populations, and the results showed that the prediction model had good adaptability to the population with grade III tumors, with an AUC of 0.803.

Predicting LNM is of great significance in EGC patients, especially in the choice of treatment methods. Some models have been developed to predict the possibility of LNM in gastric cancer [6, 16]. Chen et al. establish a nomogram to predict the LNM of patients with gastric cancer using some variables such as Boarrmann type, preoperative CA199 level, T stage, and N stage, with an AUC of 0.786 [17]. Eom et al. showed that the prediction performance of conventional models established based on tumor size, histological type, lymphatic blood vessel invasion, and depth of invasion was not enough. The predictive performance of the model can be significantly improved by adding some biomarkers such as CD44v6 and *α*1 catenin to these models [18]. However, most prediction models were developed using a small sample population, or without external validation and advanced gastric cancer population. Our prediction model was established based on the SEER database, and clinical practice data were used for external validation. The AUC of our model was 0.766, indicating good predictive performance. Unfortunately, our nomogram had a poor fit in the external population. Therefore, further validation in different populations showed that the nomogram had good adaptability to the population with grade III tumors, with an AUC of 0.803.

Our results showed that LNM was associated with T stage, tumor size, and tumor grade. Similar results were found in the study of Pokala et al. Tumor stage, grade, and size were independent predictors of LNM [13]. Previous studies have proposed that the T stage was the independent risk factor for LNM [19–21]. Tumor size was a risk factor for LNM in gastric cancer shown in many studies; a larger tumor size was correlated with a higher possibility of LNM [16, 22, 23]. Our results presented that the risk of LNM in patients with tumor sizes of ≥4 cm was 5.75 times higher than that in patients with tumor sizes <1 cm. Furthermore, T stage, size, and grade can be used to estimate the incidence of LNM in patients with early gastric adenocarcinoma and to help discuss the risks of different treatment modalities [13, 24].

Previous studies have shown that the prevalence of LNM in EGC patients ranges from 7.7 to 19.4% [21, 25, 26], and most patients underwent excessive surgery and suffered from morbidity [27]. In this case, pretreatment diagnosis of LNM status was very helpful to avoid the high morbidity and mortality of the lymphadenectomy caused by the overtreatment of patients [28]. Therefore, a nomogram that can predict LNM in patients with EGC has important clinical significance. A study by Pokala et al. indicated that patients with early gastric adenocarcinoma should be consulted on appropriate treatment options, and the impact of adverse oncological outcomes that may result from endoscopic treatment on surgical morbidity and quality of life related to major organ resection should be weighed [13].

We developed a nomogram to predict LNM in patients with EGC based on the SEER database and externally validated the model using clinical practice data. When the external validation data did not fit the nomogram, we conducted further validation based on different populations. This tool to predict the likelihood of LNM in EGC patients may help clinicians make surgical decisions. However, this study has some limitations. First, our external validation data did not fit the nomogram, which may be the difference between different races. Second, tumor ulceration [6, 29], lymphovascular invasion [6, 29], and lymph node involvement by endoscopic ultrasound [30] have been reported to be associated with LNM in some studies, but these data lacked in the SEER database.

## 5. Conclusion

A nomogram to predict the LNM in patients with EGC was developed based on the SEER database. Patients with higher T stage and tumor grade and larger tumor size were more likely to develop LNM. This tool can predict the possibility of LNM in EGC patients, which may help clinicians to make surgical decisions.

## Figures and Tables

**Figure 1:** Flow diagram of patients extracted from Surveillance, Epidemiology, and End Results (SEER) database and clinical data.

**Figure 2:** Receiver operator characteristic (ROC) curves and the area under the ROC curve (AUC) for the logistic regression prediction model in the training set, test set, and external validation. (a) ROC curves in the training set; (b) ROC curves in the test set; (c) ROC curves in the external validation.

**Figure 3:** Nomogram for predicting lymph node metastasis (LNM) in early gastric cancer (EGC) patients. (a) Nomogram; (b) example of the nomogram.

**Table 1:** Characteristics of all patients.

Variables	Clinical data (*n* = 494)	SEER data		
		Total (*n* = 842)	Training set (*n* = 505)	Test set (*n* = 337)
Age (years), mean ± SD	53.80 ± 10.60	69.4 ± 11.3	69.05 ± 11.76	69.80 ± 10.71

*Gender, n (%)*				
Female	218 (44.13)	357 (42.40)	214 (42.38)	143 (42.43)
Male	276 (55.87)	485 (57.60)	291 (57.62)	194 (57.57)

*T stage, n (%)*				
T1a	243 (49.19)	306 (36.34)	176 (34.85)	130 (38.58)
T1b	251 (50.81)	536 (63.66)	329 (65.15)	207 (61.42)

*Primary site, n (%)*				
Overlap	13 (2.63)	59 (7.01)	41 (8.12)	18 (5.34)
Lower	348 (70.45)	455 (54.04)	267 (52.87)	188 (55.79)
Middle	120 (24.29)	303 (35.99)	185 (36.63)	118 (35.01)
Upper	13 (2.63)	25 (2.97)	12 (2.38)	13 (3.86)

*Type, n (%)*				
Diffuse	302 (61.13)	69 (8.19)	36 (7.13)	33 (9.79)
Intestinal	16 (3.24)	700 (83.14)	424 (83.96)	276 (81.90)
Others	176 (35.63)	73 (8.67)	45 (8.91)	28 (8.31)

*Tumor size (cm), n (%)*				
1-	130 (26.32)	148 (17.58)	135 (26.73)	110 (32.64)
2-	151 (30.57)	245 (29.10)	117 (23.17)	57 (16.91)
3-	122 (24.70)	174 (20.67)	60 (11.88)	53 (15.73)
4-	57 (11.54)	113 (13.42)	101 (20.00)	61 (18.10)
<1	34 (6.88)	162 (19.24)	92 (18.22)	56 (16.62)

*Grade, n (%)*				
I	314 (63.56)	143 (16.98)	78 (15.45)	65 (19.29)
II	128 (25.91)	334 (39.67)	206 (40.79)	128 (37.98)
III	52 (10.53)	365 (43.35)	221 (43.76)	144 (42.73)

*LNM, n (%)*				
No	361 (73.08)	666 (79.10)	398 (78.81)	268 (79.53)
Yes	133 (26.92)	176 (20.90)	107 (21.19)	69 (20.47)

Note: LNM: lymph node metastasis.

**Table 2:** Difference analysis of patients with or without LNM in the training set.

Variables	Total (*n* = 505)	Non-LNM (*n* = 398)	LNM (*n* = 107)	Statistic	*P*
Age (years), mean ± SD	69.05 ± 11.76	69.41 ± 11.62	67.74 ± 12.24	*t* = 1.30	0.193
Gender, *n* (%)				*χ* ^2^ = 0.266	0.606
Female	214 (42.38)	171 (42.96)	43 (40.19)		
Male	291 (57.62)	227 (57.04)	64 (59.81)		
T stage, *n* (%)				*χ* ^2^ = 30.817	<0.001
T1a	176 (34.85)	163 (40.95)	13 (12.15)		
T1b	329 (65.15)	235 (59.05)	94 (87.85)		
Primary site, *n* (%)				*χ* ^2^ = 0.450	0.930
Overlap	41 (8.12)	31 (7.79)	10 (9.35)		
Lower	267 (52.87)	210 (52.76)	57 (53.27)		
Middle	185 (36.63)	147 (36.93)	38 (35.51)		
Upper	12 (2.38)	10 (2.51)	2 (1.87)		
Type, *n* (%)				*χ* ^2^ = 2.076	0.354
Diffuse	36 (7.13)	26 (6.53)	10 (9.35)		
Intestinal	424 (83.96)	339 (85.18)	85 (79.44)		
Others	45 (8.91)	33 (8.29)	12 (11.21)		
Tumor size (cm), *n* (%)				*χ* ^2^ = 27.052	<0.001
<1	135 (26.73)	110 (27.64)	25 (23.36)		
1-	117 (23.17)	92 (23.12)	25 (23.36)		
2-	60 (11.88)	43 (10.80)	17 (15.89)		
3-	101 (20.00)	66 (16.58)	35 (32.71)		
4-	92 (18.22)	87 (21.86)	5 (4.67)		
Grade, *n* (%)				*χ* ^2^ = 15.375	<0.001
I	78 (15.45)	72 (18.09)	6 (5.61)		
II	206 (40.79)	167 (41.96)	39 (36.45)		
III	221 (43.76)	159 (39.95)	62 (57.94)		

Note: LNM: lymph node metastasis.

**Table 3:** Univariate and multivariate logistic regression analyses of factors associated with LNM.

Variables	Univariate analysis		Multivariate analysis	
	OR (95% CI)	*P*	OR (95% CI)	*P*
Age	0.99 (0.97–1.01)	0.193	—	—

*Gender*				
Female	Ref			
Male	1.12 (0.73–1.73)	0.606	—	—

*T stage*				
T1a	Ref		Ref	
T1b	5.02 (2.72–9.26)	<0.001	3.84 (2.04–7.21)	<0.001

*Primary site*				
Lower	Ref			
Overlap	1.19 (0.55–2.57)	0.661	—	—
Middle	0.95 (0.60–1.51)	0.836	—	—
Upper	0.74 (0.16–3.46)	0.699	—	—

*Type*				
Diffuse	Ref			
Intestinal	0.65 (0.30–1.40)	0.274	—	—
Others	0.95 (0.35–2.53)	0.911	—	—

*Tumor size*				
<1	Ref			
1-	3.95 (1.45–10.75)	0.007	2.70 (0.97–7.54)	0.058
2-	4.73 (1.73–12.90)	0.002	3.07 (1.10–8.61)	0.033
3-	6.88 (2.38–19.89)	<0.001	4.73 (1.58–14.13)	0.005
4-	9.23 (3.43–24.84)	<0.001	5.75 (2.08–15.92)	<0.001

*Grade*				
I	Ref		Ref	
II	2.80 (1.14–6.91)	0.025	2.04 (0.80–5.21)	0.137
III	4.68 (1.94–11.32)	<0.001	3.19 (1.27–8.00)	0.014

Note: LNM: lymph node metastasis; OR: odds ratio; CI: confidence interval; Ref: reference.

**Table 4:** The area under the receiver operating characteristic curve (AUC) for different models.

Models	Training set	Test set
	AUC (95% CI)	AUC (95% CI)
Logistic regression	0.731 (0.682–0.779)	0.766 (0.709–0.823)
Ridge regression	0.730 (0.681–0.779)	0.740 (0.681–0.799)
LASSO regression	0.721 (0.671–0.771)	0.737 (0.676–0.797)
Elastic-net regression	0.735 (0.686–0.783)	0.749 (0.691–0.807)

Nomogram for prediction of LNM in EGC patients.

**Table 5:** The performance of the logistic regression prediction model.

Parameter (95% CI)	SEER data		External validation
	Training set	Test set	
AUC	0.731 (0.682–0.779)	0.766 (0.709–0.823)	0.625 (0.573–0.678)
Accuracy	0.588 (0.544–0.631)	0.588 (0.533–0.641)	0.617 (0.573–0.660)
Sensitivity	0.850 (0.769–0.912)	0.899 (0.802–0.958)	0.391 (0.308–0.479)
Specificity	0.518 (0.467–0.568)	0.507 (0.446–0.569)	0.701 (0.651–0.748)
PPV	0.322 (0.267–0.379)	0.320 (0.255–0.390)	0.325 (0.253–0.403)
NPV	0.928 (0.886–0.958)	0.951 (0.902–0.980)	0.757 (0.708–0.802)
Cutoff	0.1607	0.1607	0.1607

Note: AUC: the area under the receiver operating characteristic curve; PPV: positive predictive value; NPV: negative predictive value.

**Table 6:** The performance of the prediction model based on different populations.

Subgroup	Parameter (95% CI)	Test set	External validation
Gender (males)	AUC	0.793 (0.720–0.866)	0.603 (0.530–0.675)
	Sensitivity	0.919 (0.781–0.983)	0.621 (0.493–0.738)
	Specificity	0.580 (0.498–0.658)	0.571 (0.502–0.639)
	PPV	0.340 (0.248–0.442)	0.313 (0.235–0.400)
	NPV	0.968 (0.910–0.993)	0.828 (0.756–0.885)
	Accuracy	0.644 (0.573–0.712)	0.583 (0.523–0.642)

Gender (females)	AUC	0.729 (0.635–0.822)	0.673 (0.597–0.749)
	Sensitivity	0.875 (0.710–0.965)	0.358 (0.245–0.485)
	Specificity	0.441 (0.347–0.539)	0.821 (0.751–0.879)
	PPV	0.311 (0.218–0.417)	0.471 (0.329–0.615)
	NPV	0.925 (0.818–0.979)	0.743 (0.669–0.807)
	Accuracy	0.538 (0.453–0.622)	0.679 (0.613–0.740)

Age (≥65 years)	AUC	0.755 (0.688–0.821)	0.478 (0.339–0.617)
	Sensitivity	0.896 (0.773–0.965)	1.000 (0.832–1.000)
	Specificity	0.548 (0.476–0.618)	1.000 (0.937–1.000)
	PPV	0.323 (0.245–0.410)	0.740 (0.628–0.834)
	NPV	0.956 (0.901–0.986)	—
	Accuracy	0.615 (0.552–0.676)	0.740 (0.628–0.834)

Age (<65 years)	AUC	0.794 (0.681–0.907)	0.644 (0.587–0.700)
	Sensitivity	0.905 (0.696–0.988)	0.398 (0.307–0.495)
	Specificity	0.464 (0.343–0.588)	0.734 (0.680–0.782)
	PPV	0.339 (0.218–0.478)	0.357 (0.274–0.447)
	NPV	0.941 (0.803–0.993)	0.766 (0.713–0.814)
	Accuracy	0.567 (0.458–0.671)	0.643 (0.595–0.689)

Grade (I)	AUC	0.722 (0.583–0.861)	0.695 (0.635–0.755)
	Sensitivity	1.000 (0.158–1.000)	0.500 (0.395–0.605)
	Specificity	0.905 (0.804–0.964)	0.764 (0.702–0.818)
	PPV	1.000 (0.541–1.000)	0.475 (0.373–0.578)
	NPV	0.966 (0.883–0.996)	0.781 (0.720–0.835)
	Accuracy	0.877 (0.772–0.945)	0.685 (0.630–0.736)

Grade (II)	AUC	0.645 (0.540–0.750)	0.632 (0.523–0.742)
	Sensitivity	0.870 (0.664–0.972)	0.667 (0.482–0.820)
	Specificity	0.429 (0.332–0.529)	0.474 (0.370–0.579)
	PPV	0.250 (0.160–0.359)	0.306 (0.202–0.425)
	NPV	0.938 (0.828–0.987)	0.804 (0.676–0.898)
	Accuracy	0.508 (0.418–0.597)	0.523 (0.433–0.612)

Grade (III)	AUC	0.731 (0.647–0.815)	0.803 (0.606–0.999)
	Sensitivity	0.955 (0.845–0.994)	0.833 (0.359–0.996)
	Specificity	0.310 (0.221–0.410)	0.457 (0.309–0.610)
	PPV	0.378 (0.288–0.475)	0.167 (0.056–0.347)
	NPV	0.939 (0.798–0.993)	0.955 (0.772–0.999)
	Accuracy	0.507 (0.422–0.591)	0.500 (0.358–0.642)

Note: AUCarea under the curve; PPVpositive predictive value; NPVnegative predictive value.

## Data Availability

The datasets used and/or analyzed during the current study are available from the corresponding author on reasonable request.
